# Analysis of the Prevalence, Location, and Morphology of Maxillary Sinus Septa in a Northern Chinese Population by Cone Beam Computed Tomography

**DOI:** 10.1155/2022/1644734

**Published:** 2022-07-15

**Authors:** Wenjuan Wang, Ling Jin, Huabing Ge, Fengqiu Zhang

**Affiliations:** ^1^Department of General School of Stomatology, Capital Medical University, Beijing 100069, China; ^2^Department of Radiology School of Stomatology, Capital Medical University, Beijing 100069, China; ^3^Department of Periodontics School of Stomatology, Capital Medical University, Beijing 100069, China

## Abstract

**Purpose:**

The purpose of this study is to survey the prevalence and morphology of the maxillary sinus septum, which might increase the rate of maxillary sinus membrane perforation during maxillary sinus floor elevation surgery, among northern Chinese, and to further analyze the relationship between gender, age, edentulous type, and prevalence of maxillary sinus septa.

**Methods:**

The cross-sectional retrospective study was based on an analysis of Cone Beam Computed Tomography (CBCT) images of maxillary sinus which had been obtained from patients who visited radiology department of Beijing Stomatology Hospital of Capital Medical University (Beijing, China) during the period from January 2019 to December 2019. The data of demographic characteristic, prevalence, position, direction, and morphology of maxillary sinus septum were collected and further analyzed by SPSS version 25.0.1 and R version 3.5.1 software program.

**Results:**

595 patients were included in this study, and 1190 maxillary sinuses were analyzed and the incidence rate of the sinus septum was 46.9%. 399 (33.5%) sinuses had one or more septa in 279 (46.9%) patients. In addition, maxillary sinus septa incidence showed no significant differences among gender, age, and edentulous type. The segment second molar had the highest incidence rate of septa.

**Conclusion:**

In this study, a higher incidence of the maxillary sinus septum was found in the northern Chinese, and its distribution varied with its position, morphology, and direction.

## 1. Introduction

Implants are widely used in people who were completely or partial edentulous. The posterior maxilla indicates more challenging in implants, especially for those losing teeth for a long time. The reason might be bone atrophy and bone decline of the alveolar and pneumatolytic maxillary sinus are common in the distal region of the maxilla alveolar ridge under this scenario. Hence, maxillary sinus floor elevation is adopted in implants associated with the posterior maxilla area. Unfortunately, it was reported that the rate of perforation of the membrane of maxillary sinus, the common complication in maxillary sinus floor elevation which could reduce the survival rate of implants, was in the range of 3.6% to 53.9% in total [1–8].

The membrane of maxillary sinus, also called Schneiderian membrane [9], is a ciliated pseudostratified columnar respiratory membrane, with the goblet cells, columnar cells, and basal cells fixed to its basal membrane. The thickness of the membrane varies from 0.13 mm to 1.5 mm and the average is 0.8 mm [10]. The maxillary sinus floor elevation could promote bone mass and guide bone regeneration by using Schneiderian membrane as a nature barrier [11]. The perforation of Schneiderian membrane is associated with the increase of the duration and complexity of surgery and postoperative complications. The risk factors of the perforation of Schneiderian membrane include the presence, location, and orientation of maxillary sinus septa, the thickness of Schneiderian membrane, the residual height of maxillary bone, the presence of mucous retention cyst in maxillary sinus, and the presence of maxillary sinusitis.

Maxillary sinus septum was first noticed by Arthur S. Underwood; thus, it was also named Underwood septum [9]. The Underwood septum is a very thin fragile sickle-shaped bone wall at the margin of maxillary sinus stretching to the inner and outer walls [9], and it divides the maxillary sinus into smaller compartments. Its function is to act as masticatory force supporting strut during the dentate phase in life [12]. Several reports revealed that maxillary sinus septum showed significant correlation to maxillary sinus membrane perforation. The maxillary sinus septum might enhance the adhesive strength of Schneiderian membrane and therefore it might increase the risk of membrane perforation during the maxillary sinus floor elevation [13–16]. Various methods were adopted to categorize the orientations and locations of maxillary sinus septa in previous studies. As a result, they led to the difference in the prevalence of maxillary sinus septa among certain categories [9, 17–19]. The height of maxillary sinus septum also varied with the positions, sides, and population. The mean height was in a range between 1.63 ± 2.44 mm and 13.11 ± 3.82 mm [14, 18, 20–22]. More attention should be paid to the anatomy variation of maxillary sinus septa before maxillary sinus floor elevation.

Panoramic radiograph, multi-slice computed tomography (CT), and CBCT have been widely used by dentists. The two-dimensional (2D) radiographic images provided by panoramic radiograph are difficult to explain because of the overlapping of complex osseous structure. On the contrary, the multi-slice CT and CBCT can provide three-dimensional (3D) radiographic images. In addition, the CBCT is more popular in head and neck diagnosis because of its sensitive and accurate images, low price, low radiation dose, and high resolution [23, 24].

Better understanding of the structure of the maxillary sinus septum might help decrease the rate of perforation of the membrane of maxillary sinus. Previous studies have researched maxillary sinus septa in several population groups including European, American, and Southeast Asian but northern Chinese. Hence, the purpose of this study is to survey the prevalence, location, and direction of maxillary sinus septum structure among northern Chinese people, and to further analyze the relationship between gender, age and edentulous type, and prevalence of maxillary sinus septa.

## 2. Materials and Methods

### 2.1. Study Design

The retrospective study was based on an analysis of CBCT images of maxillary sinus which had been obtained from patients who visited radiology department of Beijing Stomatology Hospital of Capital Medical University (Beijing, China) during the period from January 2019 to December 2019. Although the images covered the area from the arcus superciliaris to the bottom of mandibular bone, the analyzed images involved in this study only the area from the posterior wall of the maxillary sinus to the lateral wall of the nasal cavity. The CBCT scans were made based on the following inclusion criteria: (1) no surgical procedures had been performed based on the results of CBCT before; (2) no detectable pathologies were present; (3) no orthodontic process was included; (4) both of the maxillary sinuses were entirely depicted and all of the images were clear; (5) no foreign bodies were present; and (6) the age of the all patients was older than 18 years. This study was approved by Beijing Stomatological Hospital Human Research Ethics Committee (CMUSH-IRB-KJ-PJ-2020-18) and all participants signed an informed consent agreement.

### 2.2. Imaging and Analysis

CBCT scans were obtained using a NewTom 3G (quantitative radiology s.r.l., Verona, Italy). All images were recorded at 120 kVP and 3-5 mA using a 9-inch field of view, an axial slice thickness of 0.25 mm, and isotropic voxels. The morphology, location, height, orientation, and prevalence of maxillary sinus septa were evaluated in axial, sagittal, cross-sectional, and reconstructed panoramic images while 3-dimensional reconstructions were used as necessary. The images were analyzed using NNT Viewer software.

The measurement in this study was conducted by a dentist (WJ.W) and a radiologist (L.J). To detect inter-observer variability, 10% CBCT images were randomly selected and measured by them independently. To detect intra-observer variability, these CBCT images were measured by the same observer twice with an interval of 2 weeks. Finally, all these measurements were analyzed to obtain the inter- and intra-observer reliabilities.

The following parameters were recorded: sex (male, female), age (at the time of CBCT), and status of the maxillary bone dentition (full dentition, partial dentition, or edentulous). The measurement was performed using digital calipers and only the sagittal images of the CBCT were used for measurement. Measuring the vertical dimension of the septa covered the area from the approximate base to the highest coronal portion and the septa over 3 mm were included in this study (Figure 1). Previous researchers divided the maxillary sinus into three segments; hence, the locations of septa were spatially divided into anterior, middle, and posterior regions. In this study, the locations of septa were spatially divided into five segments: segment 4 from first premolar distal to mesial, segment 5 from premolar distal to second premolar distal, segment 6 from second premolar distal to first molar distal, segment 7 from first molar distal to second molar distal, and segment 8 from second molar distal to maxillary tuberosity (Figure 2). This kind of method can more easily and clearly distinguish where the most prevalence of septa position is. Furthermore, the septa orientations were divided into 4 directions: coronal, sagittal, horizontal, and irregular direction (Figure 3).

### 2.3. Statistics

A descriptive analysis of the dataset was primarily performed and the results were expressed as mean±standard deviation. To assess intra- and inter-observer reliability, Cohen's kappa test was used for measurement repeatability of the observers. Differences in the location and prevalence of the septa among the edentulous, part dentulous, and full dentate groups and in the prevalence of the septa by gender, and in both the sinuses were tested by *X*^2^ test. *X*^2^-test was also used to evaluate the correlations among the variables, such as age, gender, the type of denture, and the presence of maxillary sinus septa. All statistical analyses were carried out using SPSS version 25.0.1 (SPSS, Chicago, Ill, USA) software and R software (version 3.5.1). *P-*values less than 0.05 were considered statistically significant.

## 3. Results

### 3.1. Investigation of the General Population

The patient population was 865 in the aggregate, but 270 of the 865 patients were excluded because their images exhibited pathologic changes or unsharp appearance. Finally, 595 patients were included in this study, in which 251 (42.2%) were male and 344 (57.8%) were female, and 1190 sinuses were analyzed. The age of the included patients was in the range of 18 to 81years with the mean age of 46.1 years and median age of 46 years. Patients were categorized into 4 groups according to age range ≤30 years, 31-45years, 46-60 years, and>60 years, and the proportion of each group was 15.3% (*n* =91), 32.9% (*n* =196), 33.9% (*n* =202), and 17.8% (*n* =106), respectively. Furthermore, depending on the type of dentition, all the included patients were divided into full dentition (*n* =271, 45.5%), partial dentition (*n* =312, 52.4%), and edentulous (*n* =12, 2%).

### 3.2. Detection of Maxillary Sinus Septum Incidence Rate

A total of 595 CBCT scans that fulfilled the inclusion criteria were included in this study and 1190 maxillary sinuses were observed. Maxillary sinus septa were detected in 279 patients and 595 CBCT images were analyzed. At least one septum was detected in 279 (46.8%) patients and in 399 (33.5%) maxillary sinuses. 33.3% septa were found in the right maxillary sinuses and 33.9% in the left maxillary sinuses. With regard to male patients, 127 (50.6%) showed one septum and 73 (29.1%) showed two or more maxillary sinus septa in the CBCT images. For female patients, 152 (44.2%) showed one septum and 82 (23.8%) showed two or more maxillary sinus septa in the CBCT images. In the 595 CBCT images representing 1190 single maxillary sinuses, one septum was detected in 288 sinuses (24.2%), two septa were detected in 92 sinuses (7.7%), three septa were detected in 15 sinuses (1.3%), and four or more septa were detected in 4 sinuses (0.3%). Therefore, one or more septa were detected in total 399 (33.5%) sinuses. But there were only 3 septa that completely divided the sinuses into two or more compartments (Figure 4). The distribution of patients according to the gender, the age, the side of the sinuses, the dentition type, the presence or absence, and the number of septa is shown in Table 1.

### 3.3. Orientation, Location, and Height

Of the 399 septa, 243 (46.6%) were coronally oriented (5.9% on the first premolar, 16.1% on the second premolar, 12.2% on the first molar, 42.0% on the second molar, and 23.8% on the wisdom teeth), 42 (8.0%) sagittally oriented, 60 (11.5%) transversally oriented, and 177 (33.9%) irregularly oriented. In this study, only the heights of the septa which started from the bottom of maxillary sinus were measured and their locations were recorded. The mean height of the septa was 9.66 ± 7.54 mm with the maximum value of 33 mm (complete septa). The locations of septa were spatially divided into five segments: segments 4, 5, 6, 7, and 8. The results of septum locations and the mean septum height are shown in Table 2.

### 3.4. Intra- and Inter-Observer Reliability and Correlations between Septum Incidence Rate and Other Variables

The inter-observer reliability by Cohen's kappa test was 0.93 and the intra-observer reliabilities were WJ.W: 0.93, L.J: 0.95. It indicates that the observation results have high reliability. Meanwhile, there was no significant difference in septum location between gender (*P* =0.085). In addition, maxillary sinus septa incidence showed no significant differences among gender, age, and edentulous type, and the results were listed in Table 3.

## 4. Discussion

### 4.1. Incidence Rate

Previous studies indicated that the incidence of maxillary sinus septa is various and the range of prevalence is from 26.5% to 69% [8, 9, 14, 17–22, 25–27]. The incidence of maxillary sinus septa is affected by many factors. The first factor is the change of observation methods. In decades, the observation methods for the maxillary sinus septa have been improving. In the early years, the skull of the cadaver was studied and then 2-dimensional imaging (panoramic radiography) emerged. In recent years, 3-dimensional imaging has been being widely used in head and neck examination and it is in the process of replacing multi-slice CT with Core-Bean CT. CBCT allows researchers to have clearer and more accurate images; thus, more realistic number of septa could be detected. As a result, the incidence of maxillary sinus septa increases. In fact, after the application of CBCT, the prevalence of septa increases from 1/3 to 2/3 in recent two decades. The second factor is the sample size. Previous studies indicated that with the increase of the simple size, the prevalence of septa increased. The third factor is the variety of criteria of septa. The bony prominences with a height between 2 and 4 mm were defined as septa [21]. However, some researchers defined the bony prominences with the height more than 2 mm as maxillary sinus septa and others defined the bony prominences with the height more than 2.5 mm as maxillary sinus septa [18, 20, 25–28]. Different criteria could lead to different incidence rate. In addition, races and countries of population may also affect the incidence of maxillary sinus septa.

### 4.2. Location

In this study, the new method divided the sinus into five compartments as mentioned in foregoing and it was easy to reveal the prevalence of septa in every region. The results showed that 42% of the analyzed septa were in segment 7, and it was significantly higher than those in the other segments (5.9% in segment 4, 16.1% in segment 5, 12.1% in segment 6, and 23.9% in segment 8). The results suggest that dentists may pay more attention in segment 7. The previous studies showed that the location of the septa was related to the perforation of sinus membrane in maxillary sinus floor elevation [16]. Clarifying the location of the septa before operation could help dentists to determine the difficulty of the operation better, to select the appropriate surgical procedure, and furthermore to reduce the possibility of maxillary sinus membrane perforation. There were no consistent conclusions on septa location in the previous literatures. The maxillary sinus was usually divided into three parts: anterior, middle, and posterior [29, 30]. Some researchers found that the anterior maxillary sinus had the highest incidence rate of septa [17, 29], while others believed the middle area and posterior area had it [30]. The reason for their different conclusions was that they used different methods to divide the sinus. See the details in Table 4.

### 4.3. Orientation and Height

In early studies, the directions of the maxillary sinus septa were divided into three categories, namely, coronal, sagittal, and horizontal directions. These studies showed that the coronal septa had higher incidence rate than other orientations [26–28]. In recent studies, septa were divided into 4 directions: coronal, sagittal, horizontal, and irregular because some maxillary sinus septa curved. In this study, the coronal direction had the highest incidence (46.6%), irregular direction took the second place (33.9%), and sagittal and horizontal directions were less (8.0% and 11.5%, respectively).

Bony prominences with the height between 2 mm and 4 mm were defined as maxillary sinus septa [21]. The perforation rate of maxillary sinus membrane was significantly increased in the presence of 3-6 mm septa in maxillary sinus floor elevation [13]. In this study, sinus septa were defined as bony prominence above or equal to 3 mm in height. The maximum height of septa was 33 mm, which was completely through the sinus. When there was such septum, surgeons should pay more attention on the selection of surgical methods and procedures.

### 4.4. Statistics

This study revealed that the maxillary sinus septum incidence rate was higher in man compared to women, however without significant difference which was consistent with previous studies [31]. In addition, this study found that there was no significant difference in the incidence rates among different age groups. Most studies obtained the same conclusion while few others did not, and this might be the result of the difference of age categories [22].

### 4.5. Limitations and Future Expectations

Most patients in this study were full or partial dentition while others were edentulous, and this might be caused by the sampling bias in this retrospective single-center cross-sectional study. For overcoming this bias, large multicenter studies need to be conducted in the future.

## 5. Conclusion

In this study, a high incidence of the maxillary sinus septa was found, and coronal septa had the highest incidence, and the segment second molar had the highest incidence in the bottom of the maxillary sinus. Therefore, it is helpful to take CBCT imaging examination before maxillary sinus floor elevation surgery to reduce the incidence of complications such as maxillary membrane perforation.

## Figures and Tables

**Figure 1:** The height of maxillary sinus septa. A line along the approximate base of the septum to be measured was drawn, and the height of the septum was defended by the length of a line starting from this base line to its most coronal part along the septum. Septum whose height was over 3 mm was included in this study.

**Figure 2:** The location of maxillary sinus septa. (a), (b), (c), (d), (e) show the locations of maxillary sinus septa in segments 4, 5, 6, 7, and 8, respectively.

**Figure 3:** The orientation of maxillary sinus septa. (a) coronal septa; (b) irregular direction septa; (c) sagittal septa.

**Figure 4:** A complete maxillary sinus septa.

**Table 1:** Summary of septa prevalence data.

	Number of patients	Number of septa	Septum incidence rate (%)
Patients	595	279	46.9
Male	251	127	50.6
Female	344	152	44.2
Sinus			
Right	595	198	33.3
Left	595	201	33.8
Age			
≤30	91	48	52.7
≤45	196	91	46.4
≤60	202	98	48.5
>60	106	42	39.6
Dentition type			
Full dentition	271	136	50.2
Partial dentition	312	138	44.2
Edentulous	12	5	41.7

**Table 2:** Summary of the location data and height data of septa.

Dental status	Septa location						Mean septa height ± SD^*a*^				
	4	5	6	7	8	Total	4	5	6	7	8
Full dentition	8	18	14	49	24	113	5.11 ± 1.956	5.34 ± 1.607	7.55 ± 3.438	5.85 ± 2.366	6.37 ± 6.132
Partial dentition	4	15	10	35	25	89	5.88 ± 1.302	7.84 ± 6.774	8.54 ± 9.892	7.35 ± 4.116	7.57 ± 7.386
Edentulous	0	0	1	2	0	3	—	—	5.2	5.2 ± 1.344	—
Total	12	33	25	86	49	205					

a: unit is millimeter.

**Table 3:** Correlation between septum characteristics and other variables.

Correlation between septum incidence rate and other variables	*P*-value^a^
Incidence rate of septa and gender	0.122
Incidence rate of septa and age	0.292
Incidence rate of septa and dentition type	0.333

a: chi-square test.

**Table 4:** Previous classification of maxillary sinuses.

Method	Forepart	Middle part	Posterior
1	3-5	67	8-
2	1-5	67	8-
3	45	67	8-
4	45	6	7
5	5	67	8-

## Data Availability

The datasets used and/or analyzed during the current study are available from the corresponding author on reasonable request.
